# Nutrition and mental health: A review of current knowledge about the impact of diet on mental health

**DOI:** 10.3389/fnut.2022.943998

**Published:** 2022-08-22

**Authors:** Mateusz Grajek, Karolina Krupa-Kotara, Agnieszka Białek-Dratwa, Karolina Sobczyk, Martina Grot, Oskar Kowalski, Wiktoria Staśkiewicz

**Affiliations:** ^1^Department of Public Health, Department of Public Health Policy, Faculty of Health Sciences in Bytom, Medical University of Silesia in Katowice, Katowice, Poland; ^2^Department of Epidemiology, Faculty of Health Sciences in Bytom, Medical University of Silesia in Katowice, Katowice, Poland; ^3^Department of Human Nutrition, Department of Dietetics, Faculty of Health Sciences in Bytom, Medical University of Silesia in Katowice, Katowice, Poland; ^4^Department of Economics and Health Care Management, Faculty of Health Sciences in Bytom, Medical University of Silesia in Katowice, Katowice, Poland; ^5^Department of Technology and Food Quality Evaluation, Department of Dietetics, Faculty of Health Sciences in Bytom, Medical University of Silesia in Katowice, Katowice, Poland

**Keywords:** nutrition, mental health, diet, Psychology of food, eating behavior

## Abstract

Applied psychopharmacotherapy and psychotherapy do not always bring the expected results in the treatment of mental disorders. As a result, other interventions are receiving increasing attention. In recent years, there has been a surge in research on the effects of nutrition on mental status, which may be an important aspect of the prevention of many mental disorders and, at the same time, may lead to a reduction in the proportion of people with mental disorders. This review aims to answer whether and to what extent lifestyle and related nutrition affect mental health and whether there is scientific evidence supporting a link between diet and mental health. A review of the scientific evidence was conducted based on the available literature by typing in phrases related to nutrition and mental health using the methodological tool of the PubMed database. The literature search yielded 3,473 records, from which 356 sources directly related to the topic of the study were selected, and then those with the highest scientific value were selected according to bibliometric impact factors. In the context of current changes, urbanization, globalization, including the food industry, and changes in people’s lifestyles and eating habits, the correlations between these phenomena and their impact on mental state become important. Knowledge of these correlations creates potential opportunities to implement new effective dietary, pharmacological, therapeutic, and above all preventive interventions. The highest therapeutic potential is seen in the rational diet, physical activity, use of psychobiotics, and consumption of antioxidants. Research also shows that there are nutritional interventions that have psychoprotective potential.

## Background

Inherent in urbanization and the accompanying technological and cultural development, the rush of life, the pursuit of self-actualization, and the resulting overstimulation and lack of time, affect the change in eating habits and the consumption of high-calorie and processed foods (1). We can consider them as factors influencing the development of civilization diseases, important from the point of view of public health. Among them, we cannot forget about depressive and anxiety disorders that are becoming a global epidemic (2). The number of people requiring assistance from a mental health professional is steadily increasing in Poland and worldwide. According to the International Health Metrics Evaluation (IHME), at the end of 2017, 13% of the world population suffered from mental disorders (3). The Wittchen et al. study shows that mental disorders affect 38% of the European population (4). By the end of 2019, about 1.6 million people in Poland had received psychiatric treatment (5). The situation was not improved by the COVID-19 pandemic and related sanitary restrictions, which led to the isolation of many people, with feelings of insecurity, sadness, anxiety, and misinformation (6). All this has made psychological and psychiatric help the most sought-after form of health support today. There are only about 4,300 practicing psychiatrists in Poland (7). Even fewer, only 455, are practicing child psychiatry specialists (8). Statistics are believed to be better in the psychological and psychotherapeutic support sector, although public opinion is still divided about this form of support. Moreover, registers of psychologists and psychotherapists are not common. The described phenomena lead to a transformation of the psychiatric care model and mental health support. The number of people receiving psychiatric treatment is expected to increase over the next decades. The applied psychopharmacotherapy and psychotherapy do not always bring the expected treatment result (9). As a result, other interventions are receiving increasing attention. In recent years, there has been a dramatic increase in research on the effects of nutrition on mental status, which may be an important aspect of the prevention of many mental disorders, and at the same time may lead to a reduction in the proportion of people with mental disorders.

Thus, this review aims to answer the question of whether and to what extent lifestyle and related nutrition affect mental health and whether there is scientific evidence supporting the diet and mental health relationship.

The question posed in the objective can be divided into specific questions according to which this review was divided.

Q1: Are there correlations between nutrition and mental health?
Q2: Are there psychoprotective food ingredients?
Q3: Are there nutritional interventions with proven preventive potential for mental disorders?

## Review methodology

### Methodology background

The main aspect that guided the review works conducted was to look for nutritional recommendations in the cited works regarding nutrition as psychoprophylaxis and dietary management of psychiatric disorders. Unfortunately, the current state of knowledge on this topic, despite many studies, is still poor, so the authors decided to conduct a broad review of the most current knowledge in this area to identify those sources that address the described topic and gather in one place the available knowledge.

### Review procedure

The review was conducted following good practices associated with conducting similar reviews. Literature items were searched by a team of researchers (authors) along with a library staff member trained in literature searching and EBM (evidence-based medicine) and HTA (health technology assessment). A preliminary search for items consistent with the topic and purpose of the review was conducted to identify the research field. After reviewing existing data, a keyword package was selected that seemed most relevant and consistent with the review topic.

### Eligibility criteria

The primary eligibility criteria were the language of publication, years of research or review, publication status, and whether the authors were specialists in their field (or had other publications in a similar field). Regarding language, English-language articles were selected because this language seems to be universal in the scientific community. In addition, articles that were published after 2005 were included to make sure that the topic addressed was not a completely new field of research, but also to avoid very old data, because as is known from common practice, dietetics, as well as mental health expertise, are two of the most rapidly developing scientific fields. Additionally, articles were selected that were available in full-text on an open-access basis and had impact factor values.

### Search strategy

A review of the scientific evidence was conducted based on the available literature by entering sample phrases (consistent with the MeSh dictionary) with Boole operators, logical operators (and, or, not), and special characters,: “psychodietetics,” “nutripsychiatry,” “diet,” “mental health,” “lifestyle,” “body weight,” “obesity,” “depression,” “mental disorders” (and various combinations thereof) using the methodological tool of the PubMed database. The PubMed database in this regard seems most appropriate because it is a methodological tool that allows searching for articles available in multiple scientific databases (such as Medline or Embase). Its use provides the opportunity to meet all expectations from the review (transparency, clarity, comprehensiveness, focus, uniformity, accessibility, coverage of the entire topic).

### Sources selection

The literature search yielded 3,473 records, from which 356 sources directly related to the topic of the study were selected, and then those with the highest scientific value were selected according to eligibility criteria.

The accuracy, objectivity, validity, and relevance of the evidence were tested using questions consistent with the GRADE scale: Is the information reliable? Is the information free of mistakes? Has the information been properly substantiated? Is it possible to verify the information against other reliable sources? Who are the authors? Are they qualified to present information on the topic? Are they affiliated with reputable institutions working on the issue? Is the data source peer-reviewed? For what purpose was the information? Is the information an evidenced-based fact or constitutes an opinion? Is the information subject to risk? Can this risk be estimated? When was the information published? Is the information current or outdated? Is the timeliness relevant to the issue at hand? Does the information cover the entire issue? Does the information contain background data or does it explore the issue in depth? The final literature review was based on 110 sources, representing mainly scientific output after 2005 and important multicenter studies performed after 2015. The data obtained from the review are presented in descriptive and tabular form. In addition, 11 additional sources were used in preparing the background of the research problem and the theoretical introduction.

### Critical appraisal

In critically evaluating the sources, attention was paid to whether the articles appeared in peer-reviewed journals (by at least two reviewers) and whether they had an impact factor. As described above, 110 sources were eligible for final review. A limitation of the method adopted was primarily the exclusion of sources written in a language other than English. In addition, IF has many well-documented drawbacks as a research assessment tool and therefore is not the best way to evaluate the quality of individual research articles. Nevertheless, it was chosen because it is a synthetic indicator of a source’s impact on the field of science, and a journal that has it can more likely claim to be publishing credible scientific evidence. The review did not include so-called “grey literature”, i.e., literature that has not gone through the review process or that is internal to the university (theses, conference reports, government leaflets, newsletters, etc.). Despite their multiple values, these sources are characterized by a high risk of containing outdated knowledge (Figure 1).

**FIGURE 1:** A flowchart of how to proceed in selecting bibliographic sources.

### Q1: Are there correlations between nutrition and mental health?

Excess body weight is certainly an important social problem today. More than 0.7 billion people worldwide are obese, this is about 30% of the total population, and the number of obesity-related deaths is constantly increasing (10). We consume more and more processed, high-energy, and nutrient-poor foods. Consequently, we face problems of overweight and obesity with concomitant nutrient deficiencies (quantitative malnutrition) (11). Although the level of calories consumed is increasing, we are not taking in the recommended values of micro- and macroelements that play a significant role in the proper functioning of our nervous system – B vitamins, zinc, and magnesium. Additionally, we consume less fiber- and nutrient-rich vegetables and cereal products than recommended (10, 11). Superimposing smoking, limited physical activity, and harmful alcohol consumption to the above dietary patterns, adversely affect health and development of mental disorders, including depression (10). Whose nutritional prevention is well documented in the literature (12).

The antioxidant system, which has been implicated in the development of psychiatric disorders, is relevant here (13) and its proper functioning depends on the presence of nutrients in food. In addition, the concentration of brain-derived neurotrophic factor (BDNF), which is involved in plasticity and neurodegenerative processes, depends on nutrients (14). Findings indicate a reduction in the incidence of depression and suicide with a healthy eating pattern (15, 16). Randomized trials are emerging that evaluate the efficacy of dietary change as a form of treatment for depression (15–17). Selective food supplementation can be beneficial in the treatment of psychiatric disorders. Among them, compounds such as S-adenosylmethionine, *N*-acetylcysteine, zinc, and B vitamins including folic acid, and vitamin D are mentioned. Also, omega-3 unsaturated fatty acids have a wide range of effects. They participate in synaptogenesis by influencing receptor degradation and synthesis. They have an anti-inflammatory effect and inhibit apoptosis. They affect cell membrane function, BDNF action, and neurotransmitter reuptake (18). S-adenosylmethionine (SAM) is a compound formed from adenosine and methionine, which plays a key role in methylation processes. The results of studies show its antidepressant effects (19). The use of *N*-acetylcysteine influenced the effectiveness of therapy in schizophrenia, bipolar affective disorder, or trichotillomania. It has anti-inflammatory, antioxidant, and neuroprotective effects (20). Zinc deficiency, in turn, has been linked to the severity of depressive symptoms, and its supplementation included with antidepressants plays a role in mood stabilization. Zinc modulates cytokine activity and influences neurogenesis by affecting brain-derived neurotrophic factor levels (21). B vitamins play a role in the proper functioning of the nervous tissue. Folic acid (vitamin B9) deficiency has been associated with depressive symptoms and determined in subjects with mediocre responses to antidepressants (22). Low vitamin D levels were associated with a higher risk of schizophrenia and depression (23). It has been proven that vitamin D supplementation for a period of 3 months (4,000 IU/day for 1 month and 2,000 IU/day for 2 months) significantly reduced the severity of depression, irritability, fatigue, mood swings, sleep difficulties, weakness, and ability to concentrate in adolescents diagnosed with depression. This effect is supported by studies on animal models – vitamin D contributes to the plasticity of synapses, has a neuroprotective effect, supports the production of neurotrophic factors such as nerve growth factor (NGF) and regulates the function of the dopaminergic system. (24).

For the review, the results of the most important studies on the psychoprotective effects of bioactive components contained in foods (vitamins, minerals, omega-3, and more). have been collected in tabular form (Table 1).

**TABLE 1:** Review of selected studies on the psychoprotective effect of probiotics.

Source	Sample	Bioactive ingredient	Results or conclusions
Gazerani (96)	Review article – group struggling with migraine headaches	Folate in the form of folic acid – B_9_	Addition of a methyl group to DNA methyltransferase during the DNA methylation process and adequate serum homocysteine secretion levels prevent migraine headaches
Cater et al. (97); Parikh et al. (98)	Review article – neurotherapeutic properties among healthy human populations and newborns	Docosahexaenoic acid – omega-3	Stimulates neurotransmission and development of the cerebral cortex and visual organ through the blood-brain barrier. Increased neuro-efficiency of non-verbal and verbal communication processes
Parikh et al. (98)	Review article – among a population of people with nervous system conditions – depression and newborns with encephalopathy	Alpha-lipoic acid, lignans, soluble fiber, phytoestrogen – secoisolariciresinol diglucoside	Development and size of cortical cells in the prenatal and postnatal periods. Neuromodulates cognitive-behavioral behavior. Prevention against depressive symptoms in offspring and hypoxic-ischemic encephalopathy among newborns. Reduced oxidative stress parameters in the oxidation process reducing inflammation within the nervous system
Park et al. (99); Mulati et al. (100)	Depressed patients. Blinded randomized study. *N* = 40, duration – 8 weeks An obese mouse model of neuronal impairment. Blinded, randomized study. Duration – 14 weeks	Flavonoids	Improving brain-derived neurotrophic parameter (BDNF), reducing symptoms in the pathomechanism of depression. PSD-95 protein expression affects dysfunction within synapses and neurons
Mittal et al. (101)	Review article – reduction in symptoms and progression of Parkinson’s disease	Exogenous amino acid – tryptophan	Metabolic transformations to the starting compound serotonin allow to achieve regulation of the diurnal rhythm, emotional state. Participation in the metabolism of catecholamines regulating processes at the level of the brain-gut axis. Prevention in the pathomechanism of Parkinson’s disease
Fernández et al. (102); Dogan-Sander et al. (103); Godos et al. (104)	Review studies, meta-analysis of studies. Improvement of neuronal and cognitive impairment in patients with Parkinson’s disease, schizophrenia, depression	Magnesium calcium, selenium, zinc, manganese, copper, antioxidants – vitamin D, E, C, carotenoids	Reducing the mechanism of oxidative stress achieving systemic balance consequently the absence of chronic inflammation along with a decrease in CRP, IL-6, WBC indices and somato-psychological symptoms in a depressed state.
Godos et al. (104); Burton-Freeman et al. (105)	Review studies, meta-analysis of studies Improving neuronal and cognitive impairment in patients with Alzheimer’s disease, inflammation within neurons	Complex carbohydrates, eicosapentaenoic acid, amino acid – glycine, polyphenols, anthocyanins	Regulation of neuromodulator and neurotransmitter expression. Reduced activation of the hypothalamic-pituitary-adrenal axis under the influence of lower levels of endogenous stress – lower corticosterone concentrations. Proper insulin secretion and glucose ejection into cells – adequate GLUT receptor functionality. Modulation of the processes of neurogenesis, synaptic plasticity and activation of microglia in the central nervous system. Prevention of inflammation, neurodegenerative changes through inactivation of the process of oxidation of the LDL fraction, lipid peroxidation and activation of the enzymes catalase and superoxide dismutase

Source: Own compilation based on literature review.

### Q2: Are there psychoprotective food ingredients?

The gut microbiota is estimated to form a complex ecosystem containing 1,014 microorganisms. It contains 3.3 million genes and outnumbers the human genome by about 150-fold. At the same time, it is built by more than a thousand different species of microorganisms (25). The gut-brain axis describing the bidirectional relationship between the gastrointestinal tract and the central nervous system uses several communication mechanisms. Mutual exchange of information can occur *via* the autonomic nervous system and the vagus nerve (26). Many of the effects of probiotics on mental status are associated with information transmission *via* the vagus nerve (27). Results from germ-free (GF) mice cultured under sterile conditions, devoid of detectable microorganisms, demonstrate the involvement of the gut microbiota in the proper formation and function of the endocrine system by influencing the development of the hypothalamic-pituitary-adrenal axis. The response to a stress stimulus as measured by glucocorticosteroid and adrenocorticotropin levels was significantly elevated in GF mice. It was normalized after gastrointestinal colonization with the *Bifidobacterium infantis* strain (28). Additionally, stress affects the formation and diversity of intestinal microflora (29). Another link of communication is the immune system. The microbiota is involved in the proper development of the gastrointestinal mucosal immune system (30). Bacterial antigens such as polysaccharide A, lipopolysaccharides, and thymic acids shape its proper functioning (31). The microbiota also produces neurotransmitters: gamma-aminobutyric acid, butyric acid, serotonin, dopamine, and short-chain fatty acids, which can directly affect the nervous system (32).

So, can the psychoprotective effect of strains be used in nutritional intervention? It seems reasonable here to consider the possibility of implementing treatment with probiotic preparations containing selected bacterial strains that show positive effects on the human psyche. In this approach, “probiotic” is defined as living organisms that, when consumed in adequate amounts, have a beneficial effect on the functioning of the body (33). Ilya Metchnikov was awarded the Nobel Prize in 1908 for his research on probiotics. Among them, lactic acid bacteria are the most popular. Probiotics are mainly found in fermented dairy products, or pickled products (34). Prebiotics are non-digested food components whose fermentation in the gastrointestinal tract stimulates either bacterial growth or activity or affects both, leading to the development of beneficial intestinal microflora (35). Prebiotics can include ingredients such as inulin or fructooligosaccharides. Prebiotics may also have a beneficial effect by inhibiting the growth of pathogenic bacteria. Moreover, some research results show that prebiotics can reduce inflammation by modifying the composition of the microbiota (36). Synbiotics are ingredients that contain both prebiotics and probiotics. Such a constellation allows the use of synergistic effects of these preparations. In turn, psychobiotics are defined as microorganisms that are probiotics, that show positive effects in patients treated for mental disorders (37). They can often achieve their effect through the production of neurotransmitters such as gamma-aminobutyric acid, serotonin, or other substances with an effect on the cells of the nervous system such as short-chain organic acids: acetic, propionic, or butyric (36). Oral substitution of such probiotics as *Lactobacillus helveticus* and *Bifidobacterium longum* over a period of 1 month was associated with a reduction in symptoms of anxiety and depressive disorders and a reduction in stress levels as measured by the determination of cortisol levels in animal models (38). Currently, the most effective treatment of psychiatric disorders is achieved through the use of antidepressants, or antipsychotics. However, the additional use of psychobiotics to treat anxiety or depressive disorders may prove effective in the future. It is also worth noting that popular antidepressants and antipsychotics can affect the quality of gut flora and change the composition of the microbiome to a disadvantage by killing the cultures of bacteria living in the gastrointestinal tract (39).

For the review, the results of the most important studies on the psychoprotective effect of probiotics were collected in tabular form – Table 2.

**TABLE 2:** Review of selected studies on the psychoprotective effects of substances contained in food.

Source	Sample	Preparation (Bacterial strain)	Results or conclusions
**Healthy persons**			
Diop et al. (106)	Healthy adults. Blinded, randomized study. Duration – 12 weeks	Lactobacillus acidophilus Rosell-52, Bifidobacterium longum Rosell-175 (3 × 10^9^ CFU/day)	Probiotic therapy has been shown for the first time to reduce gastrointestinal complaints in people under stress: • Significant reduction in gastrointestinal symptoms compared to the placebo group; • Significant reduction in the severity of stress-induced nausea and abdominal pain.
Messaoudi et al. (37)	Healthy adults. Double-blind, randomized study. *N* = 55, duration – 30 days	Lactobacillus helveticus R0052, Bifidobacterium longum R0175 (3 × 10^9^ CFU/day)	The first study to show that administration of a psychobiotic alleviates stress-induced psychiatric symptoms: • Reduction in anxiety symptoms on the HSCL-90 scale; • Significant reduction in anxiety and depressive symptoms; • Confirmed reduction of the stress hormone cortisol in urine; • In the group of people with lower cortisol levels (less stressed), improvements in depression and anxiety scores on the PSS, HADS, and HSCL-90 scales.
**Depression**			
Wallace et al. (107)	Depressed patients who were not taking antidepressants. Blinded, randomized study. *N* = 108, duration – 16 weeks	Lactobacillus helveticus R0052, Bifidobacterium longum R0175 (6 × 10^9^ CFU/day)	After 4 weeks of taking the psychobiotic, there was a reduction in scores on the assessment scales: • Poor mood (MADRS – Montgomery-Asberg Depression Scale, QUIDS-SR16 – Quick List of Depressive Symptoms); • Stress intensity (PSQI – Sleep Quality Questionnaire); • Anhedonia (SHAPS – Scale of Perceived Pleasure); Level of anxiety (GAD-7 – Generalized Anxiety Questionnaire, STAI – State and Trait Anxiety Inventory).
Kazemi et al. (108)	Depressed patients who were taking antidepressants (sertaline, escitalopram, fluixetine, or amitriptyline). RCT study. *N* = 81, duration – 8 weeks	Lactobacillus helveticus, Bifidobacterium longum	• Decreased scores on the Beck Depression Scale (compared to the group taking placebo or the prebiotic galactooligosaccharide). • Increase serotonin production from tryptophan (decrease in kynurenine/tryptophan ratio)
Rudzki et al. (109)	Patients with depression. Double-blind RCT study. *N* = 60, duration – 8 weeks	SSRI + Lactobacillus plantarum 299v (10 × 10^9^ CFU/day)	Augmenting SSRI treatment with probiotic bacteria Lactobacillus Plantarum 299v improved cognitive performance and reduced KYN levels in MDD patients. Reduced KYN levels may have contributed to cognitive improvement in the LP299v group compared to the placebo group
Wallace et al. (107)	Patients with depression. Double-blind RCT study. *N* = 10, duration – 8 weeks	Lactobacillus helveticus Rosell-52, Bifidobacterium Longum Rosell-175 (3 × 10^9^ CFU)	Probiotics have a role in alleviating symptoms of depression
Heidarzadeh-Rad et al. (110)	Patients with depression. RCT *post hoc* analysis. *N* = 78, duration – 8 weeks	Lactobacillus helveticus Rosell-52, Bifidobacterium Longum Rosell-175 (≥ 10 × 10^9^ CFU)	Eight-week supplementation in depressed patients improved depressive symptoms, likely by increasing BDNF levels
**Alzheimer’s disease**			
Agahi et al. (111)	Alzheimer’s patients. Double-blind RCT study. *N* = 48, duration – 12 weeks	Lactobacillus fermentum, Lactobacillus plantarum, Bifidobacterium lactis, Lactobacillus acidophilus, Bifidobacterium bifidum, Bifidobacterium longum (3 × 10^9^ CFU/day)	Cognitive and biochemical indications in patients with severe AD are insensitive to probiotic supplementation. Therefore, in addition to the composition and dose of probiotic bacteria, the severity of the disease and the timing of administration profoundly affect treatment outcomes.
Akbari et al. (112)	Alzheimer’s patients. Double-blind RCT study. *N* = 52, duration – 12 weeks	200 mL/day of milk product containing Lactobacillus acidophilus, Lactobacillus casei, Bifidobacterium bifidum, Lactobacillus fermentum (2 × 10^9^ CFU/day)	Probiotic treatment had no significant effect on biomarkers of oxidative stress and inflammation, fasting glucose and other lipid profiles. The study showed that probiotic consumption for 12 weeks had a positive effect on cognitive function and some metabolic statuses in AD patients
Tamtaji et al. (113)	Alzheimer’s patients. Double-blind RCT study. *N* = 79, duration – 12 weeks	Lactobacillus acidophilus, Bifidobacterium bifidum, Bifidobacterium longum (6 × 10^9^ CFU/day) + 200 mcg selenium	Co-supplementation of probiotics and selenium for 12 weeks in AD patients improved cognitive function and some metabolic profiles
**Chronic fatigue syndrome**			
Wallis et al. (114)	Patients with Chronic Fatigue Syndrome. Open-label study. *N* = 44, duration – 6 weeks	Alternating antibiotic and probiotic therapy: Erythromycin + Lactobacillus rhamnosus (2.5 × 10^10^ CFU/day), Bifidobacterium lactis (1.5 × 10^10^CFU/day), Bifidobacterium breve (5 × 10^6^ CFU/day), Bifidobacterium longum (5 × 10^6^ CFU/day)	Specific microorganisms interact with some ME/CFS symptoms and offer the promise of therapeutic potential targeting intestinal dysbiosis in this population
**Cognitive dysfunction**			
Hwang et al. (115)	Patients with mild cognitive impairment. Double-blind RCT study. *N* = 92, duration – 12 weeks	Lactobacillus plantarum C29 (1.25 × 10^10^ CFU/day) + powdered fermented soybeans (DW2009)	DW2009 can be safely administered to improve cognitive function in people with MCI
Kobayashi et al. (116)	Patients with mild cognitive impairment. Open-label study. *N* = 27, duration – 6 months	Bifidobacterium breve A1 (2 × 10^10^ CFU/day)	Oral supplementation of B. breve A1 in participants with MCI improved cognitive function, thus suggesting the potential of B. breve A1 for improving cognitive function and maintaining quality of life in the elderly
Kobayashi et al. (117)	Patients with mild cognitive impairment. Double-blind RCT study. *N* = 117, duration – 12 weeks	Bifidobacterium breve A1 (2 × 10^10^ CFU/day)	The results of the present study suggest the safety of B. breve A1 supplementation and its potential in maintaining cognitive function in elderly people with memory impairment

Source: Own compilation based on literature review.

Factors such as genotype, intrauterine infections, developmental disorders, later traumatizing events, use of harmful psychoactive substances, and many others will influence the onset of psychiatric disorders. These factors influence not only the onset of the disorder but also its progression. Treating early conditions in psychiatry can result in a much better response to the treatment given and better functioning of patients. This fact can be particularly observed in studies on the early detection of psychotic disorders (40). Prevention in medicine, including psychiatry, requires knowledge of appropriate and useful tools that would allow detection of increased risk of mental illness and monitoring of the developing psychopathology of the disorder. McGorry et al. (41) proposed a four-stage model of the development of mental disorders. According to this model, serious mental disorders develop from high-risk states: grade 0 means the development of undifferentiated, general symptoms, such as slight anxiety, restlessness, depressive symptoms, or somatic symptoms lead to grade 1, in which types 1A and 1B can be distinguished according to their severity. Further progression of the disease results in the development of a first episode of the disorder and here we speak of stage 2, which is accompanied by persistent 7ncludims and frequent relapses. Grade 3 includes incomplete remission and regular and repeated relapses. Grade 4 in this context means treatment-resistant disorder. The worsening of a psychiatric disorder is determined by genetic and environmental factors, and it is the latter that seems to be the main target for preventive interventions in psychiatry. Some biomarkers in psychiatry are directly related to nutrition. The first of these is the hypothalamic-pituitary-adrenal axis (HPA). Reduced ability to cope with stress plays a role in the development of psychiatric disorders (42). It is known that traumatizing experiences in early childhood shape vulnerability to stress in later life (43). The normal functioning of the HPA axis is often altered in psychiatric disorders, and increased cortisol secretion is observed in affective and psychotic disorders. Additionally, antipsychotic drugs appear to decrease HPA axis activity (44–47). Furthermore, healthy individuals who were first-degree relatives of individuals with psychotic disorders were found to have HPA axis dysfunction with elevated cortisol levels (48). These studies show that the HPA axis appears to be an important biological marker of susceptibility to developing psychiatric disorders. In this context, its association with gut microbiota is not insignificant. Other potential biomarkers involved in the pathophysiology of psychiatric disorders are inflammation and oxidative stress (49). The inflammatory theory of depression development is gaining increasing attention, and elevated levels of proinflammatory cytokines are observed in depressive, psychotic, and manic states (50, 51). Elevated levels of proinflammatory cytokines occur before the onset of *de novo* disorders, suggesting their role in the genesis of these disorders (52). An increase in oxidative stress in psychotic disorders with a decrease in glutathione and antioxidant enzymes has also been observed (53). The potential effectiveness of selective cyclooxygenase-2 antagonists in the treatment of bipolar affective disorder and schizophrenia has been demonstrated (51, 54). The use of statins, which have anti-inflammatory and antioxidant properties, reduced the risk of depressive disorders (55). Polyunsaturated fatty acids are further potential biomarkers that may have applications in psychiatry. Omega-3 polyunsaturated fatty acids may play a role in the pathogenesis of affective and psychotic disorders (56, 57). Their deficiency may be present in the early stages of psychotic disorders – stage 1b. Supplementation with omega-3 polyunsaturated fatty acids reduced the risk of psychotic disorders among individuals at high risk of developing them (58).

The intestinal barrier is composed of several layers, including the intestinal microflora, mucus layer, intestinal epithelium, and elements of the circulatory, immune, nervous, and lymphatic systems. The layer of epithelial cells, mainly enterocytes connected by tight junctions, is the most important for the intestinal barrier (59). Its main function is to regulate the absorption of nutrients, electrolytes, and water from the gastrointestinal lumen into the blood or lymphatic system and prevent the penetration of pathogens from the gastrointestinal lumen. Factors such as stress, pro-inflammatory factors, dysbacteriosis of the intestinal microflora, alcohol, or antibiotics may cause excessive permeability of the intestinal barrier (60–62). Currently, the microbiota and its diversity as a trigger for generalized inflammation are gaining great importance (61) Under the influence of the impaired functioning of the barrier, the migration of bacteria from the lumen of the gastrointestinal tract occurs, which activates the cells of the immune system affecting the functioning of the immune, endocrine and nervous systems (62). It has been observed that patients with depression have elevated IgA and IgM immunoglobulins against lipopolysaccharides of the bacterial microbiome (63). The current study indicates the use of a dietary inflammatory index, which assesses the effect of the entire diet or individual dietary components on the concentration of inflammatory markers. The results of a systematic review by Chen et al. (64) indicate that a higher dietary inflammatory index is associated with an increased risk of common psychiatric disorders, including symptoms of depression, anxiety, distress, and schizophrenia. Of particular importance is the novel finding from the dose-response analysis that a 1 unit increase in the dietary inflammatory index was associated with a 6% higher risk of depressive symptoms. Similar relationships have been observed by Firth et al. (63), particularly in schizophrenia – individuals who consume more pro-inflammatory foods and less anti-inflammatory foods are more predisposed to psychiatric disorders. At this point, it is important to look at the relationship between diet and the proper functioning of the intestinal barrier. It turns out that it is not without significance in maintaining homeostasis. A diet consisting of fast food and highly processed foods is associated with increased intestinal barrier permeability (65, 66).

### Q3: Are there nutritional interventions with proven preventive potential for mental disorders?

Epidemiological studies have shown that diet impacts mental health, and intervention studies confirm this relationship (17). The challenge for “nutritional psychiatry” is to produce comprehensive, consistent, and scientifically rigorous evidence-based studies that define the role of diet and nutrients in different aspects of mental health (67–70). Overall, few randomized trials investigate the effectiveness of dietary change in mental health treatment. One intervention study to date involved a 12-week Mediterranean diet. This study reported significant improvements in mood and reduced anxiety in adults with major depression (71) More recent RCTs – HELFIMED (72) and PREDI_DEP (73) have confirmed the benefits of a Mediterranean-style diet for mental health in depression. In contrast to these studies, in the MooDFOOD RCT, multiple nutrient supplementation did not reduce episodes of major depression in overweight or obese adults with subsyndromal depressive symptoms. This study found that multinutrient supplements containing omega-3 PUFAs, vitamin D, folic acid, and selenium neither reduced depressive symptoms, anxiety symptoms nor improved health utility indices (74). Similar results regarding the lack of effect on mental state improvement were obtained in a review of the literature in the context of vitamin D (75). For omega-3 PACs, one RCT including people with mild to moderate depression found no beneficial effect of omega-3 PACs on depressive symptoms (76). No effect of folic acid supplementation in combination with vitamin B 6 and B 12 on the onset of depression was found in older men (77) and older women (78). Furthermore, Rayman et al. (79) found no effect of selenium supplementation on mood in older people. Overall, the studies available to date, do not support the use of nutritional supplementation to prevent depression.

However, many studies confirm that higher dietary quality in adulthood is associated with a reduced risk of cognitive decline (17). Additionally, the intake of antioxidant polyphenols in older adults is associated with improved cognitive ability (80–82). Another study showed that a Mediterranean diet supplemented with olive oil and nuts was associated with improved cognitive function in an older population (83).

Therefore, we undertook an analysis of diets that could potentially affect mental health such as the MIND diet, the Mediterranean diet, and the ketogenic diet.

The MIND diet is a dietary recommendation to counteract neurodegenerative brain changes and improve nervous system function. This diet is beneficial for cognitive decline in the aging process, as well as for the prevention and progression of neurodegenerative diseases, including Alzheimer’s disease (84). The MIND diet combines the principles of the Mediterranean diet and the DASH diet, which are based on a high intake of vegetables, fruits, nuts, whole grain cereal products, olive oil, fish, and seafood, and moderate consumption of dry red wine with meals (85). Studies prove the positive effects of the DASH and Mediterranean diets on other diseases such as diabetes, cancer, and obesity (86–89).

Long-term observations confirm that adherence to the Mediterranean diet reduces the risk of developing neurological disorders by up to 28% compared to the use of other diets (83). Adherence to the MIND diet was significantly associated with a lower chance of depression and psychological distress, but not anxiety, in the entire study population (90). Like the Mediterranean diet and the DASH diet, the MIND diet emphasizes natural plant-based foods and limited intake of animal and high-fat foods, especially of animal origin. However, there are some differences between the MIND diet and the DASH diet, and the Mediterranean diet. For example, leafy green vegetables and especially berries are unique components of the MIND diet that are not included in the Mediterranean and DASH diets (90). The MIND diet does not focus on a high intake of fruit, dairy products, and potatoes. Another difference between MIND and the DASH and Mediterranean diets concerns fish consumption. In MIND, individuals consuming as little as 1 portion of fish per week receive a positive result, whereas, in the Mediterranean and DASH diets, larger amounts of fish would need to be consumed to achieve a result (91). The MIND diet significantly slows cognitive decline with age (92). The Mediterranean diet has also been shown to have a protective effect on anxiety and mental stress (93).

Mental illnesses are associated with numerous metabolic disorders in the brain and co-occur with many other metabolic disorders such as obesity, diabetes, and CVD. The ketogenic diet is an evidence-based treatment for epilepsy that has been shown to have profound effects on brain metabolism and neurotransmitter function. In a ketogenic diet, as much as 80 percent of energy can come from fat. This proportion sounds like a deal-breaker for healthy eating, but it turns out that ketones formed from fats can alleviate epileptic seizures unresponsive to anticonvulsant drug therapy (83). In the case of mitochondrial epilepsy, reports on the effects of the ketogenic diet are conflicting. In a study by El Sabbagh et al. (94), no patients on a ketogenic diet achieved no significant reduction in seizure frequency epileptic seizures. In contrast, a study by Kang et al. (95) involving 14 patients showed that the use of a ketogenic diet in 10 of them reduced the frequency of epileptic seizures by more than 50%, and in 7 patients, epileptic seizures ceased. In the analysis, there were improvements in symptoms including mood, cognitive function, communication skills, energy, anxiety, and auditory and visual hallucinations (90). Other reported benefits included positive biometric changes such as improvements in lipid profile, weight reduction, positive change in blood glucose, and reduction in HbA1c. These benefits may facilitate the management of comorbidities and improve overall health and well-being (93). This highlights that advances in nutritional psychiatry are important and it will be important to replicate, refine and scale up dietary intervention studies targeting the prevention and treatment of common mental health disorders. In addition, there is an unmet need for more randomized, controlled clinical trials (118–121).

## Strengths and limitations

There is still little work in the scientific space that summarizes the major findings related to the impact of nutrition on mental health, especially, as this review does, highlighting the importance of nutrition in psychoprevention and pointing to the psychoprotective effects of nutrients. The primary limitation of the presented review of research on the relationship between diet and mental health is the plethora of studies on the topic. The plethora of studies here does not mean that they all address the issue presented in this manuscript. Much of the work that was searched and queried assumes a relationship between nutrition and the psyche, but these tend to be very superficial opinions that are not scientifically grounded. The authors are aware that in the face of such a large body of research, important reports may have been overlooked, but it should be noted that every effort was made to ensure that this review was conducted fairly, taking into account large, multi-center research projects and highlighting the major research streams in psychodietetics and nutripsychiatry.

Additionally, it was observed that in the current state of scientific knowledge, few large meta-analyses are treating the effects of food and diet on mental health. Therefore, it is difficult to discuss the effectiveness of introducing nutritional interventions among people with mental disorders or treating nutrition as the only means of prevention. Furthermore, the primary threat to interventions of this type is the difficulty in monitoring dietary patterns or intake of specific components. In addition, their absorption and metabolism are also dependent on many factors that rarely have a consistent course. Therefore, it is postulated that further research should be directed toward the creation of unambiguous dietary recommendations for mental health problems.

## Conclusion

In recent decades, the relationship between nutrition and patients’ mental status has been underappreciated, as evidenced by the lack of research conducted before the 21st century in this area of knowledge – cited in this review. In recent years, this trend has been reversed, with research in psychodietetics and nutripsychiatry gaining popularity. In the context of current changes, urbanization, globalization, including the food industry, and changes in people’s lifestyles and eating habits, correlations between these phenomena and their impact on psychological status are becoming important. Exploring these correlations creates potential opportunities to implement new effective dietary, pharmacological, therapeutic, and above all preventive interventions (Figure 2).

**FIGURE 2:** Links between nutrition and mental health.

## Author contributions

MATG: conceptualization. MATG and KK-K: investigation and methodology. KS and AB-D: data curation. MATG: writing – original draft preparation. MATG, KK-K, MARG, and AB-D: writing – review and editing. KS and AB-D: supervision. KK-K: project administration. WS: conducting an additional literature review, creating tables summarizing current knowledge of psychobiotics and psychoprotective food ingredients, and revising the work. All authors contributed to the article and approved the submitted version.
